# Decoding the Mechanism of Shixiao Powder in Treating Coronary Heart Disease Based on Network Pharmacology and Molecular Docking

**DOI:** 10.1155/2022/3756668

**Published:** 2022-07-06

**Authors:** Zuo-min Jiang, Tong Wu, Yi-tao Xue, Yan Li, Gui-hua Li, Kai Huang, Hua-jing Yuan, Meng-qi Du

**Affiliations:** ^1^Shandong University of Traditional Chinese Medicine, Jinan 250014, China; ^2^Affiliated Hospital of Shandong University of Traditional Chinese Medicine, Jinan 250014, China

## Abstract

Shixiao powder comes from the *Formularies of the Bureau of People's Welfare Pharmacies* in the Song Dynasty and consists of two herbs, Puhuang (PH) and Wulingzhi (WLZ). PH-WLZ is a commonly used drug pair for the treatment of coronary heart disease (CHD), and its clinical effect is remarkable. However, our understanding of the mechanism of treatment of CHD is still unclear. In this study, the method of network pharmacology was used to explore the mechanism of PH-WLZ in the treatment of CHD. A total of 56 active ingredients were identified from PH-WLZ, of which 93 targets of 41 active ingredients overlapped with those of CHD. By performing Gene Ontology (GO) and Kyoto Encyclopedia of Genes and Genomes (KEGG) enrichment analysis, we obtained the main pathways associated with CHD and those associated with the mechanism of PH-WLZ in the treatment of CHD. By constructing the protein-protein interaction (PPI) network of common targets, 10 hub genes were identified. Based on the number of hub genes contained in the enrichment analysis, we obtained the key pathways of PH-WLZ in the treatment of CHD. The key KEGG pathway in the treatment of CHD by PH-WLZ is mainly enriched in atherosclerosis, inflammation, immunity, oxidative stress, and infection-related pathways. Moreover, the results of molecular docking showed that the active ingredients of PH-WLZ had a good affinity with the hub genes. The results indicate that the mechanism of PH-WLZ in the treatment of CHD may be related to regulation of lipid metabolism, regulation of immune and inflammatory responses, regulation of downstream genes of fluid shear stress, antiaging and oxidative stress, and virus inhibition.

## 1. Introduction

The report on the global burden of ischaemic heart disease from 1990 to 2019 shows that, in 2019, an estimated 9.14 million people worldwide died from coronary heart disease (CHD) and an estimated 197 million people worldwide suffered from CHD. Globally, the age-standardized prevalence of CHD and the absolute number of deaths have declined over the past 30 years, but CHD mortality has declined significantly in high-income countries and remains high in low- and middle-income countries [1]. Traditional Chinese medicine has played an irreplaceable role in the treatment of various diseases in ancient times. Chinese herbal medicines and their extracts have great potential to treat various diseases, and they have also been the focus of drug research and development in recent years. A meta-analysis including 2,405 cases showed that the combined treatment of standard Western medicine and traditional Chinese medicine compounds significantly improved the overall efficacy of CHD complicated with diabetes and improved clinical indicators such as blood lipids, blood sugar, and electrocardiogram [2]. A meta-analysis of 1806 cases showed that, compared with placebo, the traditional Chinese medicine method of promoting blood circulation and removing blood stasis has a great beneficial effect on reducing the rate and degree of restenosis in stents and it is an effective and safe treatment for CHD patients after percutaneous coronary intervention [3]. PH-WLZ is a traditional Chinese medicine pair belonging to the category of promoting blood circulation and removing blood stasis and has long been used as a therapeutic drug pair for chest pain symptoms in traditional Chinese medicine. However, due to the complexity of TCM compounds, multitarget sites, and diversity of action pathways, the mechanism of PH-WLZ in the treatment of CHD is still unclear. Network pharmacology combines bioinformatics, multimodal pharmacology, network data analysis, and computer technology to explore drug-target-disease correlations by analyzing “drug-target-disease” interaction networks [4]. Therefore, to study the mechanism of action of PH-WLZ in the treatment of CHD, this study used the method of network pharmacology to explore the targets and pathways of PH-WLZ in the treatment of CHD. The flowchart of our analysis is shown in Figure 1. The research methods of this article on network pharmacology are partly borrowed from the article by Li et al. [5]. We express our respect and gratitude to these authors for their innovations and improvements in network pharmacology research methods.

## 2. Materials and Methods

### 2.1. Active Ingredients and Related Targets of PH-WLZ

HERB (https://herb.ac.cn/) is a high-throughput database established by Professor Zhao Yi and his team, integrating multiple TCM databases (including SymMap, TCMID 2.0, TCMSP 2.3, and TCM-ID) of traditional Chinese medicine and ingredients and determining the relationship between them. Therefore, we screened the chemical constituents of PH-WLZ in HERB with the keywords of “Puhuang” and “Wulingzhi.” For the obtained results, we normalized in PubChem (https://pubchem.ncbi.nlm.nih.gov/).

SwissADME (https://www.swissadme.ch/) is a website that uses computer prediction models to reveal the physicochemical properties of small-molecule compounds and to assess pharmacokinetics, drug similarity, and medicinal chemical closeness. Oral bioavailability (OB) and drug likeness (DL), two ADME-related models, are the main variables affecting drug absorption from the gastrointestinal tract. This website evaluates the gastrointestinal absorption of compounds according to the BOILED-Egg method and evaluates the drug-like properties of compounds according to five methods: Lipinski, Ghose, Veber, Egan, and Muegge. Therefore, we screened the active ingredients of PH-WLZ based on the criteria of “high” for GI absorption and “Yes” for at least three of the five drug-like properties.

We retrieved all active ingredients on 3 target prediction web servers: BATMEN-TCM (https://bionet.ncpsb.org.cn/batman-tcm/), SwissTargetPrediction (https://swisstargetprediction.ch/), and STITCH (https://stitch.embl.de/), retrieval results as active ingredient-related targets. BATMEN-TCM is an online bioinformatics analysis tool to study the molecular mechanism of traditional Chinese medicine, and we set the retrieval parameters with score ≥40 and adjusted *p* value ≤0.05. SwissTargetPrediction is an online tool designed to predict molecular targets based on the 2D and 3D structural similarity of compounds. In the SwissTargetPrediction, the species is restricted to “*Homo sapiens*” and the probability is set as no less than 0.6. STITCH 5.0 is a database of predicted interactions between known chemical molecules and proteins. The species “*Homo sapiens*” and a confidence score ≥0.6 were set as the parameters of STITCH 5.0. Finally, to make the results concise and convenient, we canonicalize gene names using the UniProt database (https://www.uniprot.org/).

### 2.2. Known Targets of CHD

To obtain disease targets, we used “coronary heart disease” as the keyword to search for the corresponding genes of CHD in different databases. The four databases and search criteria are as follows: GeneCards (https://www.genecards.org/), and the screening criterion is relevance score ≥ 40; Comparative Toxicogenomics Database (CTD) (https://ctdbase.org/), and the screening criterion is direct evidence or inference score ≥ 60; DisGeNET (https://www.disgenet.org/home/), and the screening standard is gene-disease association score ≥ 0.1; and NCBI Gene (https://www.ncbi.nlm.nih.gov/gene), and the screening criterion is species belonging to *Homo species*. The data obtained in each database were merged to obtain the final disease targets of CHD. These targets are also canonical gene names in the UniProt database.

### 2.3. Disease Target PPI Network Construction and Cluster Analysis

STRING (https://cn.string-db.org/) is a database of known and predicted protein-protein interactions (PPIs), currently containing about 24.6 million proteins from 5,090 microorganisms. In this study, potential target interactions were analyzed using STRING, setting the species as “*Homo sapiens*” with a confidence score ≥ 0.7.

A PPI network was built to visualize disease targets using Cytoscape (version 3.9.0). Interactive network topology analysis was performed using the Network Analyzer plugin. For each node in an interactive network, the degree value is an important parameter to evaluate its topological characteristics, and it measures the number of connections with other nodes and reflects the importance of the node.

Cluster analysis aims to screen out identical or similar nodes and protein complexes from complex PPI networks. Cluster analysis of disease PPI networks was performed using the MCODE plugin (version 3.9.0) in Cytoscape. A node score cutoff = 0.2, k-core = 2, maximum depth = 100, and degree cutoff = 2 were set as the filter conditions.

### 2.4. Common Targets of PH-WLZ and CHD

Using Venny 2.1 (https://bioinfogp.cnb.csic.es/tools/venny/), we intersected the active target of PH-WLZ with the target of CHD and obtained a direct target (common genes) of the active component of PH-WLZ for the treatment of CHD.

To understand the interaction between common genes, the STRING database was used to study the interaction network between proteins and to mine the core regulatory genes. In this study, potential target interactions were analyzed using STRING, the species was set to “*Homo sapiens*,” and the confidence score was ≥0.4. We used Cytoscape (version 3.9.0) to construct a visual common target PPI network and a common target active ingredient network.

The hub gene is the bottleneck gene of node connection in the network and plays an important role in the PPI network. We used the CytoHubba plugin of Cytoscape (version 3.9.0) to identify the hub genes, and the top 10 genes generated by the maximum neighborhood component (MCC) method were regarded as hub genes. A visualized TCM-active ingredient-hub gene-disease network was constructed using Cytoscape (version 3.9.0).

### 2.5. GO and KEGG Pathway Enrichment Analysis

Gene Ontology (GO) annotation was used to define and describe the function of gene products from three aspects, namely, biological processes (BPs), cellular components (CCs), and molecular functions (MFs). The Kyoto Encyclopedia of Genes and Genomes (KEGG) is a database integrating genomic, chemical, and systemic functional information. To obtain more accurate GO and KEGG functional enrichment information, the ClusterProfiler software package of the R platform was used for GO and KEGG functional enrichment analysis, and the screening criterion was adjusted *P* ≤ 0.05. GO and KEGG pathway enrichment analysis was performed on the genes and common genes of the top 5 clusters of disease-gene cluster analysis, respectively.

The results of the disease enrichment analysis and the results of the common gene enrichment analysis were combined to obtain the GO and KEGG enrichment analysis results related to the treatment of CHD by PH-WLZ. The intersection entries contain entries with more hub genes as key results.

### 2.6. Validated with Molecular Docking

The crystal structures of the hub targets were downloaded from the RCSB PDB (https://www.rcsb.org/) database, and the structures of the active ingredients were obtained from the PubChem database. Before molecular docking, we use AutoDock (version 4.2.6) software to remove ligands, remove water molecular structure, and add hydrogen atoms and charges to the protein crystal structure. Molecular docking was performed using AutoDock Vina (version 1.1.2) software to evaluate the interaction between the target and the active ingredient. Results were analyzed and plotted using PyMOL (version 2.5.2).

## 3. Results

### 3.1. Active Ingredients and Related Targets of PH-WLZ

A total of 114 components of PH and 39 components of WLZ were retrieved from the HERB database. Among them, 26 components were not matched in PubChem and were eliminated. Based on the screening of the SwissADME platform, 71 components that did not meet the oral bioavailability or drug-like properties were eliminated, and 56 active components of PH-WLZ were obtained, including 3 repeating components of PH and WLZ. Details of these components and reasons for exclusion are listed in Supplementary Table 1.

We obtained 468, 142, and 105 targets corresponding to active ingredients in the BATMEN-TCM, STITCH, and SwissTargetPrediction databases, respectively. The intersection of the predicted targets of the three databases is shown in Figure 2(a). After removing duplicate information, a total of 42 active ingredients and 633 potential targets were obtained. See Supplementary Table 2 for gene names after UniProt database normalization.

### 3.2. Known Targets of CHD

The occurrence and development of CHD is a complex process involving the regulation of multiple genes and proteins. By screening CTD, NCBI Gene, GeneCards, and DisGeNET, we obtained 197, 271, 358, and 368 target genes, respectively. The intersection of target genes in each disease database is shown in Figure 2(b). A total of 807 nonrepetitive genes were merged, and the gene names after UniProt database canonicalization are shown in Supplementary Table 3.

### 3.3. Disease Target Analysis

Using the STRING database online service platform, the protein-protein interaction network analysis of disease target genes was performed, and the results are shown in Figure 3(a). The nodes in the middle are closer to red, and the larger the area is, the greater the representative degree value is. The largest 10 node genes are TNF, AKT1, STAT3, IL6, TP53, CTNNB1, MAPK3, EGFR, FN1, and IL1B. They play an important role in the occurrence and progression of CHD.

The PPI network of CHD targets was then clustered using the MCODE plugin in Cytoscape. Thus, 31 clusters were obtained (Supplementary Table 4). Based on their scores, we selected the top 5 clusters (Figure 3(b) and Table 1) and performed GO functional enrichment and KEGG pathway analysis on the targets covered by the 5 clusters. Finally, 2820 BPs, 73 CCs, 197 MFs, and 172 KEGG pathways were obtained (*P* ≤ 0.05). The top 10 meaningful terms in BPs, MFs, and CCs and the top 20 meaningful KEGG pathways are shown in Figures 4(a) and 4(b), respectively.

GO enrichment analysis showed that the biological processes related to CHD were mainly related to the regulation of cytokines and adhesion factors, cell proliferation, and response to foreign bodies, such as positive regulation of cytokine production, response to lipopolysaccharide, smooth muscle cell proliferation, and positive regulation of cell adhesion. CHD-related molecular functions are mainly related to binding activity and catalytic activity, such as cytokine binding to receptors, signal receptor activator activity, lipoprotein particle receptor binding, and enzyme activator activity. CHD-related cellular components are mainly related to lipid particles and cell membranes, such as high-density lipoprotein particles, triglyceride-rich plasma lipoprotein particles, membrane rafts, and membrane microdomains. KEGG pathway analysis showed that the main signalling pathways related to CHD were lipid and atherosclerosis, human cytomegalovirus infection, cytokine-cytokine receptor interaction, and PI3K-Akt signalling pathway.

### 3.4. Common Target Analysis

By comparing the targets of PH-WLZ and CHD, we found that CHD and active ingredients share 93 targets in common (Figure 5(a)), and 93 targets are related to 41 active ingredients (Supplementary Table 5). The common target-active ingredient network is shown in Figure 5(b). Based on the degree value, we identified 5 active ingredients with degree value > 8, namely, quercetin (HBIN041495), adenine (HBIN012217), naringenin (HBIN036366), palmitic acid (HBIN029268), tyramine (HBIN047435), and gallic acid (HBIN027030).

To explore the mechanism of PH-WLZ in the treatment of CHD, we used the ClusterProfiler package of the R platform to perform KEGG and GO functional enrichment analysis on 93 common targets. Therefore, we obtained 1829 BPs, 175 MFs, 107 CCs, and 159 KEGG pathways (*P* ≤ 0.05). The top 10 meaningful terms in BPs, MFs, and CCs and 20 meaningful KEGG pathways are shown in Figure 6.

GO enrichment analysis showed that the biological processes involved in common targets were mainly related to the response to stimuli, the regulation of blood vessels, and the regulation of inflammation, such as the response to exogenous stimuli, vascular processes in the circulatory system, and regulation of inflammatory responses. The main molecular functions of common targets are oxidoreductase activity, tetrapyrrole binding, heme binding, nuclear receptor activity, ligand-activated transcription factor activity, etc. Cell components are mainly in membrane rafts, membrane microdomains, plasma membrane rafts, caveola, postsynaptic membranes, etc. The most prominent pathways of common targets are chemical carcinogenesis-receptor activation, lipids and atherosclerosis, Alzheimer's disease, estrogen signalling, AGE-RAGE signalling in diabetic complications, fluid shear stress, atherosclerosis, etc.

To obtain the common target PPI network, 93 common targets were first imported into the STRING database, and the online service platform of the STRING database was used to analyze the protein-protein interaction network of the common targets; and the results are shown in Figure 7. The obtained PPI network was then imported into the Cytoscape platform, and using the CytoHubba plugin, the first 10 nodes in the network generated by the MNC method were regarded as hub genes (Figure 7(a)), namely AKT1, CASP3, CCL2, CXCL8, INS, JUN, MMP9, PTGS2, SERPINE1, and TNF. The hub gene may be the key target of PH-WLZ in the treatment of CHD. The PPI network of 10 hub genes has 10 nodes and 45 edges, the average node degree is 9, and the *P* value is 7.41*e* − 09 (Figure 7(b)).

### 3.5. Selection and Analysis of GO and KEGG Results

After comparing and analyzing GO and KEGG results for disease targets and common targets, we found 1490 overlapping BPs, 46 overlapping CCs, 74 overlapping MFs, and 136 overlapping KEGG pathways (Supplementary Table 6).

The hub gene of PH-WLZ may play a key role in the treatment of CHD. Therefore, we selected the GO and KEGG entries containing the most hub genes for further analysis. Finally, we obtained 3 key biological processes (number of hub genes ≥5), 4 key molecular functions (number of hub genes ≥3), and 2 key cellular components (number of hub genes ≥3). The key biological process of PH-WLZ treatment of CHD: response to a molecule of bacterial origin (GO:0002237), response to lipopolysaccharide (GO:0032496), and response to tumor necrosis factor (GO:0034612). Key molecular functions: cytokine receptor binding (GO:0005126), signalling receptor activator activity (GO:0030546), receptor ligand activity (GO:0048018), and cytokine activity (GO:0005125). Key cellular components are in membrane rafts (GO:0045121) and membrane microdomains (GO:0098857).

We summarized the KEGG pathways containing hub genes ≥6 and obtained 6 key KEGG pathways. Although the number of hub genes enriched in fluid shear stress and atherosclerosis and MAPK signalling pathways is less than 6, they are important CHD-related pathways [6, 7]. Eight key KEGG pathways are mainly related to atherosclerosis, inflammation, immunity, oxidative stress, and infection, as shown in Table 2. The key KEGG pathway enrichment results and the connection with key targets are shown in Figure 8.

### 3.6. TCM-Active Ingredient-Hub Gene-Disease Network

A TCM-active ingredient-hub gene-disease network was constructed based on the active ingredients related to the hub genes (Figure 9). This network has 32 nodes (2 herbs, 19 active ingredients, 10 hub genes, 1 disease) and 56 edges. PH has the most active components acting on the hub gene and plays a major role in PH-WLZ. Based on degree values and references, we found gallic acid (HBIN027030), isorhamnetin (HBIN031114), quercetin (HBIN041495), kaempferol (HBIN031753), and naringenin (HBIN036366) in the crown, which play an important role in CHD and atherosclerosis. They may be the key active components of PH-WLZ in the treatment of CHD.

### 3.7. Validated by Molecular Docking

According to the TCM-active ingredient-hub gene-disease network, we treat the connected hub targets and key active components as receptors and ligands, respectively. The stability of receptor and ligand binding depends on the binding energy. The lower the binding energy, the more stable the binding conformation of the receptor and ligand. We set a binding energy of −5.0 kcal/mol as the threshold for determining whether receptor and ligand binding is good. The interaction of receptor and ligand is shown in Figure 10. As shown in Table 3, all active ingredients can bind well to the central target.

## 4. Discussion

CHD is characterized by atherosclerosis in the coronary arteries, leading to blockage of the vascular lumen and subsequent myocardial ischaemia, hypoxia, and necrosis. The formation of atherosclerotic plaque (As) is the pathological basis of CHD, and its occurrence and development are a chronic inflammatory process involving multiple steps and factors. AS is a multifactorial disease involving chronic inflammation, lipid metabolism and accumulation, oxidative stress, genetic predisposition, immune disorders, epigenetics, and multiple nongenetic risk factors (environmental pollution, smoking, mental health, diet, and lifestyle). The “multiple hits” hypothesis suggests that all these injuries work together to cause atherosclerosis.

Through constructing PPI network of PH-WLZ and CHD, common targets, AKT1, CASP3, CCL2, CXCL8, INS, JUN, MMP9, PTGS2, SERPINE1, and TNF found to be the hub genes of PH-WLZ in the treatment of CHD. These genes are mainly associated with atherosclerosis, inflammation, immunity, oxidative stress, and infection. Based on the analysis of hub genes, key active components, and major prominent KEGG pathways, the underlying mechanism of PH-WLZ in the treatment of CHD may be attributed to the following aspects.

### 4.1. Regulate Lipid Metabolism

Arterial narrowing by lipid-rich plaques in the arterial vessel wall is a major feature of atherosclerosis, and elevated low-density lipoprotein (LDL) cholesterol levels are a major risk factor for atherosclerosis. LDL can accumulate in blood vessel walls and be modified by oxidation to form oxidized LDL (oxLDL). OxLDL causes endothelial cell dysfunction, inducing the expression of adhesion molecules and the recruitment of monocytes in the subendothelial space. Monocytes proliferate, differentiate into macrophages, and take up lipoproteins to form cholesterol-rich “foam cells.” Lectin-like oxidized low-density lipoprotein receptor-1 (LOX-1) mediates the recognition and internalization of oxLDL, acting on multiple cells, such as endothelial cells, macrophages, platelets, fibroblasts, and smooth muscle cells; it plays a central role in atherosclerosis [8]. PIK3CA and AKT1 in the intersection targets are the key components of Akt-PI3K pathway, which is an important signal transduction pathway downstream of LOX-1. AKT has serine/threonine kinase activity and can be activated by phosphorylated Akt (p-Akt) under the action of PI3K. And p-Akt further activates downstream factors of function involved in apoptosis, protein synthesis, metabolism, and cell cycle substrates to control key cellular processes. Phosphorylation of AKT activates the 3B isoform of cyclic nucleotide phosphodiesterase (PDE3B), resulting in decreased cyclic AMP levels and inhibition of lipolysis [9]. Phosphorylation of AKT can potentially regulate ATP-citrate lyase (ACLY activity) and thus regulate fatty acid synthesis [10]. Of course, lipids including low-density lipoproteins, very low-density lipoproteins, and their oxides have inflammatory effects and participate in the process of inflammatory response [11], which will be described separately later.

### 4.2. Regulate Immune and Inflammatory Responses

In recent years, atherosclerosis has been regarded as a chronic inflammatory disease, which is an abnormal response of the vascular wall to various injuries, and has the characteristics of classic inflammatory degeneration, exudation, and proliferation. Inflammatory response runs through all stages of atherosclerosis and may be a common link or pathway in the pathogenesis of various atherosclerotic factors. The immune and inflammation-related pathways in the results included IL-17 signalling pathway, TNF signalling pathway, and MAPK signalling pathway.

The interleukin 17 (IL-17) family is a subgroup of cytokines composed of IL-17A-F, which plays an important role in the inflammatory response of autoimmune diseases, as well as injury, physiological stress, and infection [12]. The IL-17 family signals through its corresponding receptors and activates downstream pathways including TAK1, NF-kappa B, MAPK, and TNF to induce the expression of antimicrobial peptides, cytokines, and chemokines [13]. However, we checked the enrichment of the intersection genes in the IL-17 signalling pathway and found that the intersection genes were mainly enriched in the middle and lower reaches, especially in the pathways associated with the TNF signalling pathway and the MAPK signalling pathway, and no upstream IL-17 family members were found in the intersection genes. Therefore, the role of PH-WLZ in regulating immunity and inflammation may be mainly related to the downstream TNF signalling pathway and MAPK signalling pathway.

Tumor necrosis factor (TNF) is a key cytokine that induces a wide range of intracellular signalling pathways, including apoptosis and cell survival as well as inflammation and immunity. Activated TNF assembles into homopolymers and binds to its receptors (TNFR1, TNFR2). TNFR1 signalling induces the activation of many genes, including the NF-kappa B pathway and the MAPK pathway; and TNFR2 signalling activates the NF-kappa B pathway, including the PI3K-dependent NF-kappa B pathway and the JNK pathway [14]. Studies have confirmed that the TNF-mediated NF-kappa B pathway can increase endothelial inflammation and significantly increase the degree of atherosclerotic lesions [15]. We observed that AKT1, CASP3, CCL2, JUN, MMP9, PTGS2, and TNF in key genes all appeared in the TNF signalling pathway, and many were in key positions in the pathway. Therefore, the inflammatory mechanism mediated by the TNF signalling pathway may be the most critical inflammatory mechanism of PH-WLZ in the treatment of CHD.

The MAPK signalling pathway is a cascade reaction composed of a series of protein kinases and their phosphorylation. The activation of MAPK is involved in the regulation of the inflammatory response in AS. In general, ligands as inflammatory substances first activate the corresponding receptors, which in turn activate the MAPK molecules, which subsequently lead to the activation of the transcription factor NF-KAPPA B, thereby regulating the expression of inflammatory cytokines [16]. Experiments have shown that by adding the MAPK inhibitor U0126, the levels of MAPK and NF-kappa B were downregulated, and the content of atherosclerotic plaques and macrophages in mice was significantly reduced [17].

### 4.3. Regulation of Downstream Gene Activation by Fluid Shear Stress

Atherosclerosis preferentially occurs in tortuous regions, branch points, and bifurcations of the arterial tree due to endothelial dysfunction caused by the action of nonlaminar characteristic fluid shear stress, which activates the expression of endothelial-related genes. Endothelial dysfunction leads to the activation of downstream signalling pathways including AP-1, NF-kappa B, Akt-PI3K, and MAPK, and the expression of these genes promotes the oxidative and inflammatory state in the arterial wall, which leads to the occurrence of atherosclerosis [18]. The AP-1 dimer transcription complex family refers to dimeric transcription factors consisting of Jun, Fos, or ATF (activating transcription factor) subunits that associate with a common DNA site (the AP-1 binding site) combined and involved in almost all cellular and physiological functions. Studies have confirmed that activated c-Jun/AP-1 signalling can promote the proliferation and migration of vascular smooth muscle cells, while in atherogenic apolipoprotein E-deficient (ApoE−/−) C57BL/6 mice with high fat in a dietary atherosclerosis model, interference with TRIM7 can effectively alleviate atherosclerosis in vivo by inactivating the c-Jun/AP-1 signalling pathway [19]. Akt-PI3K and MAPK signalling pathways have been mentioned above, and the results show that stable liquid shear stress activates the mechanosensor platelet endothelial cell adhesion molecule-1 (PECAM-1), resulting in phosphorylation of PI3K, which in turn activates integrins. Following activation by alpha-fatty hormone, focal adhesion kinase (FAK) is phosphorylated, resulting in downstream phosphorylation of MAPK p38. Then, phosphorylation of MAPK signalling leads to COX-2 mRNA transcription, post-transcriptional COX-2 protein synthesis, and release of PGI2, an important antiatherosclerotic prostaglandin [18].

### 4.4. Fights Aging and Oxidative Stress

Atherosclerosis is considered a distinct disease of biological and cellular aging that promote premature or accelerated vascular aging under cardiovascular risk factors [20]. The AGE/RAGE signalling pathway is considered highly associated with aging, oxidative stress, and certain pathological conditions such as hyperglycemia, and activation of the AGE-RAGE axis triggers the occurrence and progression of atherosclerosis [21]. Intracellular hyperglycemia promotes the production of mitochondrial reactive oxygen species (ROS) and increases the formation of intracellular advanced glycation end products [22]. Activation of AGE/RAGE triggers the activation of multiple intracellular signalling pathways involving NADPH oxidase, protein kinase C, PI3K-Akt, and MAPKs, followed by NF-kappa B activity [23]. NF-kappa B promotes the expression of proinflammatory cytokines (such as IL-1, IL-6, and TNF-*α*) and various atherosclerosis-related genes (including VCAM-1, tissue factor, VEGF, and RAGE) [24]. Among the common targets, AGTR1, NOX4, PIK3AC, NOS3, MAPK1, JUN, and CASP3 occupy important positions in the AGE/RAGE signalling pathway.

### 4.5. Virus Suppression

Many infections are thought to be associated with CHD, such as HIV, human, cytomegalovirus, *Chlamydia pneumoniae*, *Helicobacter pylori*, etc. The inflammation and immune response brought about by infection activate or accelerate the process of atherosclerosis. Human cytomegalovirus infection is significantly associated with CHD and coronary atherosclerosis [25]. In the context of low immunity, human cytomegalovirus infects endothelial cells, resulting in endothelial cell damage and altered metabolism, and then infects smooth muscle cells, leading to proliferation and accumulation of cholesterol and cholesteryl esters. And the latent infection is repeatedly activated, causing repeated damage to the arterial wall. In infected cells, aberrant apoptotic changes may play an important role in pathogenesis [26]. Although the hepatitis B-related pathway is one of the key results, recent studies have shown that HBV infection does not increase the risk of CHD [27]. Therefore, in some viral infection-related CHD, the active ingredients of PH-WLZ may play a role.

### 4.6. Research on Key Active Ingredients

Gallic acid is a phenolic acid widely distributed in many different families of higher plants with high antioxidant properties. Gallic acid can improve high glucose levels, insulin, inflammation, and oxidative stress in diabetic complications by activating multiple effective pathways such as NO/iNOS generation, AGE/ALE, and JNK/ERK [28]. The anti-inflammatory mechanism of gallic acid mainly involves the MAPK and NF-kappa B signalling pathways, which attenuate the inflammatory response by reducing the release of inflammatory cytokines, chemokines, adhesion molecules, and cellular infiltration [29]. In addition, in an experimental diabetic rat model, oral administration of gallic acid significantly reduced serum total cholesterol, triglycerides, and LDL-cholesterol [30].

Isorhamnetin, naringenin, kaempferol, and quercetin are all flavonoids, and many studies have shown that these flavonoids have a wide range of pharmacological activities, including antioxidant, anti-inflammatory, antibacterial, anticancer, cardioprotective, neuroprotective, antidiabetic, etc. These flavonoids also have extensive preventive and therapeutic effects on cardiovascular and cerebrovascular diseases, such as antiatherosclerosis, protection of endothelial cells, antimyocardial ischaemia, antihypotension, antihypoglycemia, and antithrombosis. Isorhamnetin can protect cardiovascular cells from inflammation, oxidative damage, and apoptosis by affecting PI3K/AKT, NF-kappa B, and MAPK signalling pathways [31]. Naringenin can directly or indirectly regulate cytokines such as TNF-*α*, IL-6, IFN-*γ*, and signalling pathways NF-kappa B and MAPK and has a relieving effect on atherosclerosis [32]. Kaempferol-induced upregulation of GPER attenuates atherosclerosis through the PI3K/AKT/Nrf2 pathway [33]. Quercetin prevents the development of atherosclerosis in ApoE−/− mice by regulating the expression of PCSK9, CD36, PPAR*γ*, LXR*α*, and ABCA1 [34].

## 5. Conclusion

We obtained the key active ingredients of PH-WLZ in the treatment of CHD, namely, gallic acid, isorhamnetin, quercetin, kaempferol, and naringenin, and these active ingredients are mainly derived from PH. By constructing a compound-target-disease network, 10 hub genes were screened, namely, AKT1, CASP3, CCL2, CXCL8, INS, JUN, MMP9, PTGS2, SERPINE1, and TNF. We obtained meaningful biological processes, molecular functions, cellular components, and KEGG pathways by performing GO and KEGG pathway analysis. The results of key active components, hub genes, and enrichment analysis indicated that the mechanism of PH-WLZ in the treatment of CHD may be related to the regulation of lipid metabolism, regulation of immune and inflammatory responses, regulation of downstream gene activation caused by fluid shear stress, and antiaging and oxidative stress, and virus inhibition.

## Figures and Tables

**Figure 1:** Flowchart of exploring the mechanism of PH-WLZ in treating CHD. The active ingredients of PH-WLZ and their potential targets were predicted from different databases. The relevant targets of CHD were collected from four different databases. The intersections of the active ingredient targets and disease targets were regarded as common targets. The pivotal active ingredients were obtained through a common target-active ingredients network analysis. The overlapping pathways were obtained through pathway enrichment analysis of the disease targets and common targets. We used the CytoHubba plugin to select hub genes in the common targets. Finally, the pivotal active ingredients, overlapping pathways, and hub genes were analyzed to explore the mechanisms of PH-WLZ in treating CHD. The one-way arrow indicates the relationship of progressive research paths, and the two-way arrow indicates the relationship of intersections.

**Figure 2:** Number of targets collected in major databases and their intersection. (a) Target prediction results of drug active ingredients: a total of 633 nonrepetitive targets were collected from the three compound target prediction sites, and only 6 were shared across the three databases. (b) Collected disease targets: a total of 807 disease targets were collected from four databases, of which 49 targets were shared by the four databases.

**Figure 3:** Protein-protein interaction (PPI) network and cluster analysis of the disease targets. (a) PPI networks of CHD targets. The node in the middle that is closer to red and larger in area represents the larger degree value. (b) Top five clustering graphs from the PPI network of CHD targets.

**Figure 4:** Gene Ontology (GO) and Kyoto Encyclopedia of Genes and Genomes (KEGG) analysis of CHD-related genes. (a) Top 10 significantly enriched terms in biological processes (BPs), cellular components (CCs), and molecular functions (MFs). (b) The 20 pathways with the lowest *q* values. The *X*-axis is the GeneRatio of the term, and the *Y* axis is the name of the terms. The darker the color, the smaller the *q*value. The larger the circle, the greater the number of target genes in the term.

**Figure 5:** Common target and common target-active ingredient network. (a) Common target of PH-WLZ and CHD. (b) Common targets-active ingredients network. Blue nodes represent the common targets of CHD and PH-WLZ; purple nodes represent the active ingredients of PH related to the common targets; and red nodes represent the active ingredients of WLZ related to the common targets.

**Figure 6:** Gene Ontology (GO) and Kyoto Encyclopedia of Genes and Genomes (KEGG) analysis of common targets. (a) Top 10 significantly enriched terms in biological processes (BPs), cellular components (CCs), and molecular functions (MFs). (b) The 20 pathways with the lowest *q*-values. The *X*-axis is the GeneRatio of the term, and the *Y*-axis is the name of the terms. The darker the color, the smaller the *q*value. The larger the circle, the greater the number of target genes in the term.

**Figure 7:** Identification of hub genes of PH-WLZ for CHD. (a) Ninety-three common target protein-protein interaction (PPI) networks. This network has 91 nodes and 916 edges. (b) PPI network of hub genes.

**Figure 8:** Hub targets and key KEGG pathway. The left curve connects the relevant hub targets to key KEGG pathways. The *X*-axis of the bubble diagram on the right is the GeneRatio of the term, and the *Y*-axis is the name of the terms. The darker the color, the smaller the *q*-value. The larger the circle, the greater the number of target genes in the term.

**Figure 9:** Disease-hub gene-active ingredient-herb network. Triangle nodes represent disease, arrow-like nodes represent hub genes, circle nodes represent the active ingredients related to the hub genes, the square nodes represent herbs, and the diamonds nodes represent disease. The size of the nodes was set according to their degree value.

**Figure 10:** Molecular docking of key active ingredients on hub genes.

**Table 1:** TOP5 cluster information of the CHD protein-protein interaction (PPI) network.

Cluster	Score	Nodes	Edges	Gene symbols
1	16.606	34	274	IFNG, LCAT, APOC3, APOE, APOA1, IL18, CD4, APOB, CETP, HP, CXCL10, TLR2, IL10, APOA5, CCL3, APOL1, IL2, APP, CLU, IL17A, APOA2, APOC2, IL15, APOC1, IL7, IL1A, APOA4, CCL2, LPA, PLA2G7, CXCL8, APOC4, PON1, IL4
2	14.941	52	381	MPO, ALB, MYC, TNNT2, TLR4, ESR1, TP53, MAPK3, BDNF, NFKB1, IL1R1, TNF, MMP9, PTEN, HRAS, CRP, CAV1, PTGS2, MTOR, CCR5, KRAS, MYBPC3, SHC1, MYL2, STAT3, SMAD4, SOS1, IL7R, POMC, JUN, CTNNB1, FOS, CTLA4, MMP3, BCL2L1, VCAM1, CD40LG, ERBB2, ACTN2, CCR2, MYH6, LEP, IRS1, IGF1, TTN, TPM1, SIRT1, AKT1, TNNI3, ICAM1, PTPN11, CASP3
3	7.86	58	224	TGFBR2, GSTP1, HPGDS, MAPK1, IRAK1, CASP1, KDR, ITGB3, TGFB3, RELA, CYP2C19, HIF1A, CYP3A4, AGTR2, CREB1, CYP2C9, TWIST1, IL33, IL6, NLRP3, TNFRSF1A, CXCL12, IL6R, FGFR1, STAT1, HTR2C, SMARCA4, TGFB2, ESR2, CDKN2A, SELP, CYP2C8, ADRB2, IL23R, CDKN1A, BRCA1, GSK3B, IL22, EZH2, SELE, CYCS, CASP9, SMAD2, ATM, CYP1A1, TGFB1, CYP1A2, EPHX1, IL1RN, VEGFA, TGFBR1, TSC2, NFKBIA, FGF2, IL1B, SMAD6, CX3CL1, GSTM1
4	5	5	10	CYBA, NCF1, NCF2, CYBB, NOX4
5	5	9	20	SLC30A8, FTO, LRP5, LRP6, CDKAL1, KCNJ11, TCF7L2, APC, IGF2BP2

**Table 2:** Results of key KEGG analysis.

Classification	ID	Description
Atherosclerosis	hsa05417	Lipid and atherosclerosis
	hsa05418	Fluid shear stress and atherosclerosis
Inflammatory and immune	hsa04668	TNF signalling pathway
	hsa04010	MAPK signalling pathway
	hsa04657	IL-17 signalling pathway
Oxidative stress	hsa04933	AGE-RAGE signalling pathway in diabetic complications
Infection	hsa05163	Human cytomegalovirus infection
	hsa05161	Hepatitis B

**Table 3:** Screening docking results between ligands and receptors.

Hub targets(PDB ID)	Active ingredients	Binding affinity (kcal/mol)
MMP9 (1GKC)	Quercetin	−10.4
PTGS2 (5F19)	Isorhamnetin	−8.1
CCL2 (7SO0)	Naringenin	−7.0
PTGS2 (5F19)	Gallic acid	−6.5
JUN (5T01)	Gallic acid	−6.2
AKT1 (1H10)	Isorhamnetin	−6.1
AKT1 (1H10)	Quercetin	−6.0
MMP9 (1GKC)	Kaempferol	−5.9
SERPINE1 (1A7C)	Gallic acid	−5.9
CASP3 (1CP3)	Gallic acid	−5.7

## Data Availability

The data used to support the findings of this study are available from the corresponding author upon request.
